# Synergistic Antitumor Activities of Docetaxel and Octreotide Associated with Apoptotic-Upregulation in Castration-Resistant Prostate Cancer

This article has been retracted.

**DOI:** 10.1371/journal.pone.0091817

**Published:** 2014-03-14

**Authors:** Sha Zhu, Judith Apondi Oremo, Sanqiang Li, Minghui Zhen, Yue Tang, Ying Du

**Affiliations:** 1 Department of Microbiology and Immunology, College of Basic Medical Sciences, Zhengzhou University, Zhengzhou, P. R. China; 2 Department of Biochemistry and Molecular Biology, Medical College, Henan University of Science and Technology, Luoyang, P. R. China; UC Davis Comprehensive Cancer Center, United States of America

## Abstract

Androgen deprivation therapy has become the fist-line treatment of metastatic prostate cancer; however, progression to castrate resistance disease occurs in the majority of patients. Thus, there is an urgent need for improvements in therapy for castration-resistant prostate cancer. The aims of the present study were to determine the efficacy somatostatin analogue octreotide (OCT) combined with a low dose of docetaxel (DTX) using castration resistant prostate cancer cells and to investigate the involved molecular mechanisms in vitro. The anti-proliferative and synergism potential effects were determined by MTT assay. Induction of apoptosis was analyzed employing annexing V and propidium iodide staining and flow cytometry. VEGFA, CASP9, CASP3 and ABCB1 gene expression was evaluated by RT-PCR and Q-RT-PCR analysis. OCT in combination with DTX treatments on DU145 cell migration was also evaluated. Investigation revealed that combined administration of DTX and OCT had significant, synergistically greater cytotoxicity than DTX or OCT treatment alone. The combination of the two drugs caused a more marked increase in apoptosis and resulted in greater suppression of invasive potential than either individual agent. There was obvious increase in caspase 3 expression in the OCT alone and two-drug combined treatment groups, however, VEGFA expression was markedly suppressed in them. These results support the conclusion that somatostatin analogues combined with docetaxel may enhance the chemotherapy efficacies through multiple mechanisms in castration-resistant PCa cell line. This work provides a preclinical rationale for the therapeutic strategies to improve the treatment in castrate resistance disease.

## Introduction

Prostate cancer (PCa) is the most common cancer which represents a great threat to men's health. Androgen deprivation therapy (ADT) involving surgical or chemical castration is the standard treatment for patients with advanced PCa [1]. However, most patients will become refractory to androgen deprivation and ultimately progress with castration-resistant diseases [2], usually within 12–24 months from initiation of hormonal therapy [3]. The emergence of aggressive castration-resistant clones during ADT is rationale for taxane-based therapy, which is the only chemotherapy class to show a survival benefit in metastatic castration resistant prostate cancer (CRPC) [4], [5].

Docetaxel (DTX) is the first-line chemotherapeutic option for symptomatic CRPC patients who are candidates for chemotherapy [6], which enhances the overall response, clinical remission of the prostate cancer patients [7]. DTX treatment increases Bcl-2 phosphorylation, down-regulates Bcl-XL protein levels, induces p53 and thus results in apoptosis [8], [9]. In addition, DTX was reported to exert antiangiogenic effects [10]. It reminds us of the early evidence that taxotere could inhibit the proliferation of human umbilical vein endothelial cell proliferation through inhibition of VEGF secretion [11]. Therefore, we investigated VEGFA secretion before and after treatment with various agents. However, cytotoxicities especially peripheral neurotoxicity and hematopoietic side-effects are significant and inevitable progression occurs after DTX treatment [12], [13]. Resistance can develop through a variety of mechanisms include inhibition of apoptosis and activation of the extracellular signal-related pI3 kinase/Akt survival pathways with the development of metastasis [14]. Due to resistance, it often fails to cure patients, therefore, it is important to identify better or alternative therapeutic strategies that reverse chemotherapy resistance and enhance sensitivity to docetaxel-based chemotherapy drugs.

Somatostatin (SST) was discovered as an inhibitor of growth hormone which was first isolated from the hypothalamus of sheep. It is distributed in many human organs and tumors with a variety of functions such as inhibition of cell proliferation, regulation of phosphotyrosine phosphatase activities to inhibit the PI3 kinase and MAP kinase activities [15]. Many synthetic somatostatin analogs (octreotide, lanreotide, vapreotide, and depreotide) were developed and five different subtypes of somatostatin receptors can be bound by them [16]. Somatostatin receptors are present on cell membranes of castration-resistant PCa cell lines, however, their dynamic expression can vary depending on the phenotypic feature of each cell line [17]. The synthetic somatostatin analog octreotide (OCT) has been extensively studied as one of the SST analogs and accumulating evidence supports its antitumor activity in cancer therapy [18], [19]. OCT has been approved by FDA to be used as a standard of care for the medical treatment in various types of cancers. It has a highly improved stability compared with natural somatostatin, allowing for long-term treatment [20].

Combing different anticancer agents is a reasonable strategy with which to obtain a potent cytotoxic effect in cancer cells. In our study, we determined the effect of combined treatment of DTX and OCT on the profile of genes expression associated with apoptosis, angiogenesis and drug-tolerance in DU-145 cells. The results presented herein showed that the association of DTX and OCT provided a more than additive apoptotic response. This novel drug combination was more efficient at inducing apoptosis and reducing migration than either drug alone. These results provide an overall understanding of the clinical strategies of prostate cancer and drug resistance reversal.

## Materials and Methods

### Cells and cell culture

DU145 prostate cancer cells and PC3 cells were provided kindly as a gift by Prof. Peter Nelson (Fred Hutchinson Cancer Research Center). They are purchased from the American Type Culture Collection (ATCC, Manassas, VA, USA). The cells were cultured in Dulbecco's Modified Eagle Medium (DMEM, Invitrogen, Carlsbad, USA) that was supplemented with 10% fetal bovine serum (FBS) (Hyclone) and 1% penicillin/streptomycin at 37°C in a humidified atmosphere with 5% CO2. Confluent cells were passaged with trypsin-EDTA (0.05% trypsin and 0.53 mM tetrasodium EDTA) and harvested to prepare mRNA as described below.

### Treatment and cell viability assay

DU145 prostate cancer cells were seeded in 96-well plates in quintuplicate with Dulbecco's basal medium plus 10% fetal bovine serum and maintained in culture for 24 h. The cells were treated with DTX (5, 10, 20, 50 or 100 nM) and OCT (10, 10^2^, 10^3^, 10^4^, 10^5^ nM), used alone or in simultaneous combinations for 24 h, 48 h and 72 h, respectively. At the end of incubations, cell medium was removed and 100 µL/well of MTT solution (0.5 mg/mL in PBS) were added. Then, plates were incubated for 3 h (at 37°C, protected from light). After incubation at 37°C, 5% CO2 for 4 h, the supernatants were removed carefully, and 150 µl of DMSO was added to each well. The cells were then shocked for 10 min in the dark. Absorbance was measured at 450 nm in a Microplate Reader (Bio-Rad 680). Analysis of the obtained results was done using GraphPad Prism 4 computer program to evaluate cell proliferation rate and cytostatic rate. Untreated cells were used as controls.

### RNA and DNA extraction

Total RNAs from cultured cells were extracted using Trizol reagent (Takara, Dalian, China) according to the manufacturer's instructions and their concentrations were determined by a spectrophotometer (NanoDrop, Nyxor Biotech). Genomic DNAs from cultured cells were extracted using DNeasy Blood & Tissue Kits (Qiagen) and their concentrations were measured with the NanoDrop Spectrophotometer. All the processes were carried out according to the manufacturers' instructions.

### RT-PCR and Q-RT-PCR

Quantitative real-time PCR was performed with the QPK-201 SYBR Green master mix (Toyobo, Osaka, Japan) and the ABI 7300 system from Applied Biosystems. The primers used in the study were obtained from Invitrogen (Beijing, China) and presented in Table 1. Thermocycling parameters included a RT step at 50°C for 20 min, followed by a DNA polymerase activation step at 95°C for 2 min and 50 PCR cycles (95°C for 20 s, 60°C for 30 s). All reactions were conducted in triplicate. The fold-change in differential expression for each gene was calculated using the comparative C_T_method (also known as the 2^−ΔΔCT^method) as described by Lu et al [21].

**Table 1:** Primers used for RT-qPCR analysis.

Objective genes	Primer sequences
CASP3	Forward: 5′-CTCATACCTGTGGCTGTGTATC-3′
	Reverse: 5′-GCTCCTTTTGCTGTGATCTTC-3′
ACBC1	Forward: 5′-GTCGGAATGGATCTTGAAGGG-3′
	Reverse: 5′-ACATCAAACCAGCCTATCTCC-3′
CASP9	Forward: 5′-AGAGATTCGCAAACCAGAGG-3′
	Reverse: 5′-CAAGATAAGGCAGGGTGAGG-3′
VEGFA	Forward: 5′-CCGAAACCATGAACTTTCTGC-3′
	Reverse: 5′-CCTTTCCCTTTCCTCGAACTG-3′
β-actin	Forward: 5′-AAGGGCCATCCACAGTCTTC
	Reverse: 5′-AGAAGGCTGGGGCTCATTG

### Flow cytometric evaluation of annexin V-FITC/PI-stained cells

Cancer cells were grown on 6-well plates for 24 h, treated with DTX (20 nM) and OCT (10^3^ nM) alone or in simultaneous combination for additional 48 h. To detect apoptotic events, cells were washed twice with PBS and the pellet was re-suspended in 1× Annexin binding buffer at a concentration of 10^6^cells/ml. Then, 100 µl of the cell suspension was transferred to 5 ml culture tube. Next, 5 µl of the Annexin V-FITC and 5 µl of Propidium Iodide were added to each test, and samples were incubated for 15 min at room temperature in darkness. After this time, 400 µl of 1× Annexin binding buffer was added to each tube and cells were analyzed using a BD FacsCanto flow cytometer (BD Biosciences). Each experiment included the control samples cells stained with Annexin V-FITC (no PI) and cells stained with PI (no Annexin V-FITC). Viable cells were Annexin V-FITC- and PI-negative, cells in early apoptosis were Annexin V-FITC-positive and PI-negative and cells in late apoptosis or dead were positive both for Annexin-FITC and PI. Results were represented as fold changes in relative mean ratios between cells untreated as compared with the different treatment modalities. Each experiment was performed in triplicate.

### Wound healing assay

The scratch assay was performed to assess the influence of DTX and OCT on prostate cancer cell motility alone and in combination. DU145 cells were seeded in a high density at 6-well plates and grown for 24 h. The medium was removed and replaced with medium containing DTX and/or OCT for another 24 h. The monolayer cells were physically wounded by scratching the surface with a pipette tip (1000 µl) as uniformly and straight as possible. The images of cells invading the scratch were captured at indicated time points (0, 4, 6, 8 and 24 hrs) using phase contrast microscopy (IX 70 Olympus Optical Co., Germany). The pictures were evaluated by measuring the difference in the area of the wounds with a Leica image analysis system (Leica, Mannheim, Germany) and migration rate expressed as percentage of scratch closure was calculated as follows: % of scratch closure = a−b/a, where (a) is a distance between edges of the wound, and (b) is the distance which remained cell-free during cell migration to close the wound. The experiments were repeated in triplicate wells at least two times.

### Statistical analysis

The data from the experiments were analyzed using the SPSS 18.0 software and expressed in the form of the mean ± SD. The two-sided Student's t-test was used to analyze the differences in the experiments. The p-value <0.05 was regarded as significant whereas p-value <0.01 or <0.001 as highly significant.

## Results

### Apoptotic properties of DU145 cells treated by DTX alone, OCT alone and their combination for 48 h

In the initial study, the growth inhibitory effect of DTX, OCT and the combination of them on prostate cancer cells DU145 was examined. Following these agents treatment, parts of the cells start to shrank, inter-cell spacing became larger and cytoplasmic particle deposition was observed in the DTX and OCT treated cells. This effect was much more powerful in the combination treatment group than in the individual treatment groups. There were more floating and foaming cells displayed morphological features of apoptosis in the combination treatment groups and the increase in the treatment concentration enhanced the apoptotic appearances. Fig. 1 shows the cell morphology of different concentrations of DTX and/or OCT treatment for 48 h. In addition, as the treatment time progressed, cell growth became slow and there were increased numbers of floating cells can be observed in the medium.

**Figure 1:** Comparison of the morphology of DU145 cells treated with DTX, OCT alone and the two-drug combination for 48 h. A. Untreated cells; B. 1 nM DTX; C. 100 nM OCT; D. 10 nM DTX; E. Two-drug combination of 10 nM DTX and 100 nM OCT; F. 100 nM DTX.

### Growth inhibition by DTX and OCT alone respectively

The growth inhibitory effect of DTX and OCT was examined respectively. It is obvious that each of the two agents displayed anti-proliferation effect on DU145 cells (Fig. 2A and 2B). Both DTX and OCT decreased cell proliferation in a time and dose dependent manner. As shown in Fig. 2C, compared with untreated controls, there were 14%, 31% and 43% inhibition in the proliferation of DU145 cells exposed to 10 nM of DTX at 24 h, 48 h and 72 h. As for OCT (Fig. 2D), compared with the control, the there was a 10%, 18% and 29% inhibition in the proliferation of DU145 cells exposed to 100 nM of the drug at 24 h, 48 h, and 72 h. Data showed that the highest cytotoxicity was at 72 h and IC_50_ values of DTX (Fig. 2A) and OCT (Fig. 2B) were calculated from cell proliferation plots respectively. DTX exhibited a stronger cytotoxity with the lower IC_50_ with a value of 10.784±3.122 nM than the OCT showed a weaker inhibition effect with IC_50_ being 2.342±0.262 µM.

**Figure 2:** Inhibition of cell growth by different concentrations of DTX (A), OCT (B) after 72 hours incubation and in a time- and dose-dependent manner both of them respectively (C and D) on DU145 proliferation. Cell viability was determined by MTT assay and expressed as a percentage of the control value (mean ± SEM of three experiments done in triplicate); error bars = SEM (n = 6).

### DTX along with OCT produces synergistic inhibition of growth in human DU145 cells

To assess the possible synergistic effects of DTX-OCT combined on the growth of the cancer cells, DU145 cells were exposed to different concentrations of DXT and OCT combined for 72 h (Fig. 3B). The synergistic effect of DTX and OCT on DU145 cells proliferation was observed. The percentages of cell growth inhibition induced by DTX in combination with OCT were greater than each single agent alone. At the concentration of 10^3^ nM, OCT significantly reduced the IC50 value (P<0.05) and promoted apoptosis (P<0.05) in the DU145 cells in response to DTX. As shown in Fig. 3A, 10 nM DXT and 10^2^ nM OCT result in a 39% and 14% inhibition in proliferation in DU145 cells, respectively while both combined at the same doses caused a 68% decrease in cell proliferation compared with untreated control, which indicated a strong synergy.

**Figure 3:** Effect of DTX alone, synergistic effect of DTX in combination with 100(Fig. 3A) and various concentrations of two agents (Fig. 3B) on DU145 cells proliferation following 72 h of treatment. Results are the percentage of control value obtained with untreated cells (mean ± SEM of three experiments done in triplicate). (**) Proliferation was significantly decreased (*p*<0.001); error bars = SEM.

### VEGFA, CASP3, CASP9 and ABCB1 mRNA expression in DU145 cells

To explore the potential mechanism by which DTX plus OCT induces apoptotic cell death, the expression of genes involved in apoptotic signal, cell resistance to DTX and angiogenesis were evaluated by RT-PCR and qRT-PCR following 48 h (Fig. S3) and 72 h of treatment. Compared to the control, 10 nM DTX and 100 nM OCT, the two agents combination group markedly decreased VEGFA mRNA expression (Fig. 4A) (P<0.01). As for CASP9 and CASP3, the basal mRNA level of CASP9 and CASP3 were low but detectable and the mRNA expression was increased significantly as demonstrated in Fig. 4B and Fig. 4C (P<0.01). The protein expression level of the two caspase genes was also examined and consistent with the result of qRT-PCR (Fig. S4). In addition, the expression of ABCB1, which is recognized as a gene associated with drug resistance [22], was not affected in the treatment groups (Fig. 4D). These results imply that the anti-tumor effect of DTX in combination with OCT might be involved in promoting apoptosis associated with high expression of caspase 9 and caspase 3.

**Figure 4:** Effects of DTX, OCT alone and the combination of DTX/OCT on the mRNA expression of VEGFA, caspase 9, caspase 3 and ABCB1 in DU145 cells. M: Marker, The expression levels of objective genes were examined by RT-PCR (A, B, C and D) and quantitative real-time -PCR (B, D, F and H) respectively, using cells treated with the test drugs for 72 hours. The expression level of each mRNA was normalized to the level of β-actin mRNA. Values represent the means±SD of triplicate analyses (*p<0.05, **p<0.01).

### Effects of DTX, OCT alone and two-drug combination treatment on DU145 cells apoptosis

According to the qRT-PCR results, the experiments were divided into four treatment groups, including the control, DTX (10 nM), OCT (100 nM) and the two-drug combination groups (Fig. 5). Following treatment for 48 h, an apoptosis test was carried out by flow cytometry according to the instructions provided in the Annexin V-FITC/PI staining kit (Fig. 5A). In contrast to the control group, apoptosis was induced in both the DTX and OCT groups (P<0.05). Consistent with previous observations, the proportion of apoptotic cells was markedly increased by application of DTX plus OCT as compared with DTX or OCT treatment alone (Fig. 5B). These results indicate that the combination treatment enhanced apoptotic cell death in DU145 cells.

**Figure 5:** Effect of DTX, OCT alone and two-drug combination treatment on DU145 cells apoptosis. Data are mean ± SEM of two independent experiments performed in triplicate. ***p<0.000 vs. control.

### Effect of DTX, OCT alone and two-drug combination on the migration of the DU145 cells

To detect the effect of the two-drug combination on the migration of DU145 cells, a wound healing assay was performed following 24 h treatment. The results of the wound healing assays showed that either of the drug alone have the inhibitory effect on cells migration. But the cells in the combination group migrated more slowly than those in the drug alone and untreated control groups (Fig. 6A). Compared with the control, the relative migrated distance of the cells in the DTX, OCT and DTX/OCT combined groups (Fig. 6B), respectively were 76.5±10.21, 53.2±12.13, 79.4±13.04 (P<0.05). The cells incubated in the control group migrated across an area that was markedly larger than that of the cells incubated in the drug-combined group, indicating that DTX in combination with OCT inhibited the migration of the DU145 cells.

**Figure 6:** Effects of DTX, OCT alone and two-drug combination on DU145 cells migration. (A) Wound healing assay to determine the effect of indicated drugs on DU145 cells migration. (B) The summarized migration ratio (%) following 72 h treatment measured by wound healing assay. Each column represents the mean ± SEM. **p<0.01, vs. control.

## Discussion

Microtubule-targeting based chemotherapy is the most widely used method in the treatment of prostate cancer [23]. However, long-term treatment often results in side effects and chemotherapy resistance, usually contributing to the variable clinical outcomes among patients with seemingly similar tumor types. In an attempt to overcome drug resistance, we decided to investigate the effective cytotoxic and apoptotic concentrations of the microtubule-targeting drug docetaxel (DTX) and somatostatin analogue octreotide (OCT) and their synergistic effect of the two drugs in castration resistant prostate cancer cell line DU145.

In this study, we evaluated the combined effect of DTX and OCT against prostate cancer DU145 and PC3 cells (Fig. S1). The combination of DTX with OCT induced a greater decrease in cell viability than either agent alone. OCT reduced the IC_50_ value of DTX in DU145 and PC3 cells in a dose-dependent manner, inhibited PCa cells proliferation (Fig. S2), increased DTX sensitivity, cellular cytotoxic and apoptosis. Although we found that PC3 cells showed more sensitive to DTX than DU145 cells which consistent with the study in vivo (Fig. S5). These results suggest that OCT synergistically potentiates the efficacy of microtubule-targeting agents in PCa cells in vitro. These consistent with the recent study by Lattanzio et al. docetaxel combined with octreotide synergistically enhanced the effect of combined treatment in a particularly docetaxel-resistant PC-3 cell line [24]. However, we found either of the two drugs alone stimulates proliferation of DU145 cells in a lower concentration of DTX<1 nM or OCT<10 nM respectively, which was not observed in their combined group.

The anti-proliferative effect of DTX and OCT may be due to either cell necrosis or cell apoptosis. Therefore we investigated the apoptotic effect of DTX, OCT alone and their combination treatment in DU145 cells. Results showed that the combination of DTX with OCT decreased cell viability and increase caspase 9/3 activity to a greater extent than either single agent alone in a time dependent manner (Fig. S4). Compared with the control there is obvious increase in caspase 3 expression particularly in the OCT alone and two-drug combined treatment groups. This is consistent with the report showed that OCT increased the caspase 3 mRNA expression and induced cell apoptosis in HepG2 cells [18]. It was indicated that apoptotic programme of cell death was fired by activating the initiator caspase-8, inducing mitochondrial outer membrane permeabilization (MOMP), mitochondrial fragmentation, and ultimately activation of the downstream proteases caspase-9 and -3. MOMP induced the exit of cytochrome c, the formation of apoptosome and ultimately activation of caspase-9 [25]. In the present study, Caspase 9 activity was significantly increased after treatment of DU145 cells after the combination of DTX and OCT treatment, implicating the MOMP and mitochondrial fragmentation induction, resulting in the observed activation of apoptosis in the DU145 cell line.

VEGF signaling promotes angiogenesis by stimulating vascular endothelial cell proliferation, migration and tube formation and markedly increases vascular permeability [26]. The VEGF family includes five members, VEGF-A, VEGF-B, VEGF-C, VEGF-D and placental growth factor (PlGF) and VEGF-A is known for its key roles in tumor-related angiogenesis [27]. Therefore, we investigated the effect of OCT, DTX and the combination of the two drugs on VEGFA expression in DU145 cells. Study showed that the combination of DTX and OCT exert a great inhibitory effect on VEGFA mRNA expression but had a moderate effect by DTX alone treatment. Report demonstrated that VEGF expression was significantly suppressed in glioma cells by OCT dose-dependently. However, OCT had little effect in the microenvironment of hypoxia-induced VEGF production in vivo [28].

In the present study we demonstrated a significant decrease in cell migration in vitro after exposure to the two-drug combination treatment. Study suggests that DTX in combination with OCT inhibits DU145 proliferation or migration through inhibition of release of the peptide VEGFA and subsequently results in the inhibition of the cell migration. Study reported that the increase of VEGF/VEGFR interaction enhances the migration of colon cancer cells [29]. However, some inconsistent study results were discovered. For example, in Hepatic ischemic-reperfusion injury model, OCT showed the inhibitory effect on hepatocellular apoptosis and attenuated hepatocyte damage caused by ischemic-reperfusion [30]. Short-term application of OCT could induce OCT receptor SSTR2 desensitization and internalization, which inhibited the apoptotic effect of OCT in liver cancer cells [31]. These contrary results may be due to the different cell characteristics, cell microenvironment, expression of the receptors and OCT treatment concentration.

It is reported that ABCB1 is expressed in over fifty percent of drug-resistant cancers and recognized as a main mechanism underlying drug resistance [32]. ABCB1 expression was up-regulated after chemotherapy in various tumors as a generalized stress response [33], [34]. In our study no significant difference was noted among the various groups treated with combined DTX and OCT, each single agent alone and the untreatment control. High expression of ABCB1 gene before and after these drugs treatment indicates a DTX and/or OCT drug resistant cell line of prostate cancer DU145 cells which has been observed in our previous study by mouse xenograft model in vivo (data not published).

These data suggest that combined treatment of DTX and OCT in DU145 and PC3 cells exerted a greater inhibition of tumor cell proliferation and markedly induced apoptosis, which may be related to the up-regulation of caspase 9/3 activity and decreased expression of VEGFA in vitro. Although our results need to be extended to in vivo models in future studies, they raise the intriguing possibility that targeting microtubules with a taxane combined a somatostain analogue may be a useful approach to improving outcomes in prostate cancer.

## Supporting Information

Figure S1 **Effect of DTX alone, synergistic effect of DTX in combination with 100 nM OCT on PC3 cells proliferation following 48 h (A) and 72 h (B) of treatment.** Results are the percentage of control value obtained with untreated cells (mean ± SEM of three experiments done in triplicate). (**) Proliferation was significantly decreased (*p*<0.001); error bars = SEM.
(TIF)

Figure S2 **Synergistic effect of DTX in combination with OCT on DU145 cells proliferation following 48 h of treatment.** Results are the percentage of control value obtained with untreated cells (mean ± SEM of three experiments done in triplicate). (**) Proliferation was significantly decreased (*p*<0.001); error bars = SEM.
(TIF)

Figure S3 **Effects of DTX alone, OCT alone and the combination of DTX/OCT on the expression of VEGFA, caspase 9, caspase 3 and ABCB1 in DU145 cells by qRT–PCR respectively, using cells following 48 h of treatment.** The expression level of each mRNA was normalized to the level of β-actin. Values represent the means±SD of triplicate analyses (*p<0.05, **p<0.01).
(TIF)

Figure S4 **Detection of caspase 3, and caspase 9 expression in DU145 cells by western blot (A).** Results show that significantly increased caspase 3 and caspase 9 expression levels in DTX alone and in combination with OCT following 48 h treatment. (B) Densitometric analysis was performed using Kodak one-dimensional image analysis software. (p<0.01).
(TIF)

Figure S5 Growth curves of prostate cancer xenograft PC3 (A) and DU145 (B) in control mice, castrated mice and mice treated with docetaxel including two groups of 10 mg/kg and 20 mg/kg docetaxel treatment. Tumor measurement starts from the drug treatment (p<0.015). (n = 5).
(TIF)
